# Level Set Image Feature Detection and Application in COVID-19 Image Feature Knowledge Detection

This article has been retracted.

**DOI:** 10.1155/2023/1632992

**Published:** 2023-05-17

**Authors:** Dongsheng Ji, Yafeng Liu, Qingyi Zhang, Wenjun Zheng

**Affiliations:** ^1^School of Computer and Communication, Lanzhou University of Technology, Lanzhou 730050, China; ^2^Information Engineering University, Lanzhou 730050, China; ^3^Lanzhou Yuanchuang Electromechanical Technology Co., Ltd., Lanzhou 730030, China

## Abstract

Artificial intelligence (AI) scholars and mediciners have reported AI systems that accurately detect medical imaging and COVID-19 in chest images. However, the robustness of these models remains unclear for the segmentation of images with nonuniform density distribution or the multiphase target. The most representative one is the Chan-Vese (CV) image segmentation model. In this paper, we demonstrate that the recent level set (LV) model has excellent performance on the detection of target characteristics from medical imaging relying on the filtering variational method based on the global medical pathology facture. We observe that the capability of the filtering variational method to obtain image feature quality is better than other LV models. This research reveals a far-reaching problem in medical-imaging AI knowledge detection. In addition, from the analysis of experimental results, the algorithm proposed in this paper has a good effect on detecting the lung region feature information of COVID-19 images and also proves that the algorithm has good adaptability in processing different images. These findings demonstrate that the proposed LV method should be seen as an effective clinically adjunctive method using machine-learning healthcare models.

## 1. Introduction

In the segmentation method based on image region features, the region information fidelity parameters are used to optimize the region homogeneity, and the fidelity parameters of statistical variance are often used for continuous iteration to obtain the homogeneity of the target region [1]. The Mumford-Shah (MS) model is the most influential and mature split system. The minimization of the MS function results in a segmented image very similar to the target, which is infinitely close to the original target [2], with minimal boundary length and minimal shape difference from the original target. Therefore, there are many methods that combine image edge and regional feature information [3].

The CV model is a special form of MS model, the set *K* is represented as the boundary Γ, and the image *u*_0_(*x*, *y*) is separated by Γ. The region *Ω* in (*x*, *y*) is the two subdomains, the inner boundary Γ and the outer boundary Γ. The minimal form of the CV model can be expressed as

(1) $$\begin{array}{c} F{\left(c_{1},c_{2},\Gamma \right)}_{\text{CV}}=\lambda_{1}\int_{\text{inside}\left(\Gamma \right)}{\left|u_{0}-c_{1}\right|}^{2}dx+\lambda_{2}\int_{\text{outside}\left(\Gamma \right)}{\left|u_{0}-c_{2}\right|}^{2}dx+\mu \text{length}\left(\Gamma \right), \end{array}$$

in which *c*_1_ and *c*_2_ are the average intensities of the inner and outer boundaries of Γ, respectively. *λ*_1_ > 0, *λ*_2_ > 0, *μ* ≥ 0 are all fixed parameters, and the parameter *μ* controls the size of the detection target. *λ*_1_ and  *λ*_2_ control the driving force of the corresponding inner and outer contours of image data [4].

Although, the CV model is nonconvex and it has been widely used in the field of image segmentation. If the image intensity is close to the piecewise constant, then many special problems can be solved successfully [5]. However, if the initial assumption is exceeded and the CV model is extended to meet the requirements of image segmentation, such as the segmentation of heterogeneous images. It creates a situation where the image features are missed or some of the target boundaries are not processed [6]. However, the detection effect of the model is better, and the boundary separation between the target and the background region is more accurate. In the practical application of medical image detection, it is expected that the CV model can not only segment the homogeneous target region well but also completely determine the target feature structure and has a good segmentation of heterogeneous images [7, 8]. The constant intensity multiphase flow image detection model has acquired many types of redundant boundary information in the target, even though the segmentation is complete, while the spilt accuracy is reduced because many details are ignored in an image [9, 10]. After analysis, based on the study of the CV model, this paper proposes an extended algorithm model called the global feature filter variational minimization level set (LS) model. This algorithm can detect medical image feature targets with low contrast, nonuniform pixel intensity, noise, and multisegment boundary, and the robustness of the models remains clear for the segmentation image.

## 2. Active Contour Model (ACM)

The CV model can be improved in many aspects in the current research achievements [11]. Common thoughts mainly include the following: one is to study the role and effect of the driving force of image curve evolution and the other is to use different image fidelity terms to study from the perspective of image gradient information. The improved algorithm of the CV model is described from different research perspectives [12, 13].

The classic CV model detects the detectable phenomenon of heterogeneous images and multisegmented target images, while the variational segmentation model can quickly capture the target of interest features in an image [14, 15]. The specific situation will be explained and analyzed in the following part.

### 2.1. Local Active Contour Model (LACM)

The variational improved CV segmentation model can process the image feature with uneven intensity distribution, but its ability to process the details of the target image is still insufficient [16]. But, the LACM combined with the local area information knowledge of the image, it uses a new image information fidelity term:

(2) $$\begin{array}{c} \int_{\text{inside}\left(\Gamma \right)}{\left(u_{0}^{*}-u_{0}-d_{1}\right)}^{2}dxdy+\int_{\text{outside}\left(\Gamma \right)}{\left(u_{0}^{*}-u_{0}-d_{2}\right)}^{2}dxdy. \end{array}$$

The *u*_0_^∗^(*x*, *y*) = *g*_*k*_∗*u*_0_(*x*, *y*) is defined as the smoothing function of the image. The LS model of the local CV energy function is expressed as

(3) $$\begin{array}{c} F\left(u=1_{\Omega_{c}},c_{1},c_{2},\lambda \right)=\int_{C}g\;ds+\lambda \int_{\Omega }\left({\left(u_{0}-c_{1}\right)}^{2}-{\left(u_{0}-c_{2}\right)}^{2}\right)1_{\Omega_{c}}dxdy, \end{array}$$

in which *g*_*k*_ is the average curvature operator of the *k* × *k* image size window and *u*_0_^∗^(*x*, *y*) is used to process noise in the image. The first regularization term ∫_*Ω*_*δ*_*ε*_(∅)|∇∅|*dxdy* of the energy function keeps the target contour evolution curve smooth. The second term of the energy function is a measure to ensure the level set function *ϕ* close to the distance function in the image domain *Ω*. ∫_*Ω*_(*u*_0_ − *c*_1_)^2^*H*_*ε*_(*ϕ*)*dxdy* + ∫_*Ω*_(*u*_0_ − *c*_2_)^2^*H*_*ε*_(*ϕ*)*dxdy* is the global fitting term which guides the active contour in capturing the main structure of the image target.

Compared with the CV model, the local minimization active contour model (LMACM) has better performance in processing low noise or heterogeneous intensity image targets, and the LMACM has a better ability in capturing small details and detecting heterogeneous information than the CV model [17, 18]. However, when there is high intensity noise in the target, the method will process the noise in the image as the segmentation target, resulting in a lot of unnecessary segmentation information.  Figure 1 is the segmentation effect of low-noise and heterogeneous images. In Figure 1(b), the CV model didn't entirely detect all the boundaries and details of the image. In Figure 1(c), LACM completely detected the boundary of the target image, and the boundary is relatively smooth and without leakage on segmentation. The LACM has stronger anti-noise ability and better ability to capture target boundary information than the common CV model.

### 2.2. Global Active Contour Model (GACM)

When the comparison is very low between the image background and segmentation, the processing capacity of the CV model is limited by the locality principle [19]. The GACM based on the global feature combines the excellent capability of the CV model and global minimization of the active contour [20]. The main idea of the global feature minimization model is as follows.

First, the length of evolution curve length(Γ) in the CV model is represented as the weight term; second, new variables *u* = *H*(*ϕ*) are designed to define a convex function, where *u* ∈ {0, 1}; and it is the constraint condition on the segmentation image used to drive the convex function. Then, the minimum evolution function of the segmentation model can be expressed as

(4) $$\begin{array}{c} F\left(u=1_{\Omega_{c}},c_{1},c_{2},\lambda \right)=\int_{C}gds+\lambda \int_{\Omega }\left({\left(u_{0}-c_{1}\right)}^{2}-{\left(u_{0}-c_{2}\right)}^{2}\right)1_{\Omega_{c}}dxdy. \end{array}$$

Equation (4) is the convex function of the image *u*, where *g* = *g*(|∇*u*|), and 1_*Ω*_*c*__ represents the characteristic function. The minimization form of the variational evolution function can be expressed as

(5) $$\begin{array}{c} \underset{u,v}{\min}\left\{\int_{\Omega }g\left|\nabla u\right|dxdy+\frac{1}{2\theta }{\left\|u-v\right\|}^{2}+\int_{\Omega }\left[\lambda \left({\left(u_{0}-c_{1}\right)}^{2}-{\left(u_{0}-c_{2}\right)}^{2}\right)v+\alpha v\left(v\right)\right]dxdy\right\}, \end{array}$$

where *v*(*ξ*) = max{0, (2|*ξ* − 1/2| − 1)} and 0 ≤ *u* ≤ 1. When the LS has the fidelity term and the boundary detection function term of the image object, the model is transformed into the global minimum LS of bidirectional evolution, that is, the global minimum segmentation algorithm. The global minimization segmentation algorithm has a better image segmentation effect than the CV model, but it still has some shortcomings. In the processing of the local boundary, it still relies on the change of pixel intensity, and the ability to capture objects is not strong.  Figure 2 shows segmentation results of the images by GACM.

The global minimization optimized ACM can well process images with uniform intensity distribution. The multiphase model can also process the intensity distribution. However, if the image target has heterogeneous distributed intensity or more than two distributed intensities, neither the global minimization ACM nor the CV model can detect such an image target. The experimental effect of the global feature active contour model on MR brain images can be seen in Figure 2.  Figure 2(a) is a brain medical image; it has a complex texture structure and gray scale distribution. We can see the result from Figure 2(b), which is the experiment after 1200 times of iteration convergence, although the gray matter and the white matter of brain images have a clear break up. The algorithm can only detect part of the structure of the image and lost many feature details. This fully shows that the algorithm still lacks sufficient adaptability to the image with a certain intensity change, and it is still necessary to strengthen the study on the adaptability and detail processing ability of the target gray intensity change. In the following section, the filter image feature differentiation calculation method will be applied to further study the algorithm.

## 3. Anisotropic Diffusion Filtering Variational LS

The LS model is always maintained as a continuous binary function in the evolution process, which can well solve the problem of topological change in the evolution of the zero-level set curve without topological change of the surface [21]. The level set model only has a single data-fitting term. When the image has a heterogeneous intensity region and noise, the ability of the algorithm to segment the image is limited and the target cannot be captured effectively, which has been verified in the previous level set experiment [22].

The idea of combining global and local image structure information leads the level set model to capture small details other than noise, which can completely detect the structure information of the image target. Local image information is beneficial for the algorithm to process the target region with varying intensities, and the algorithm can completely detect the regional target structure, while the global image information can be used to detect the global structure of the image target, and the global image information combined with local area information can capture important target details except noise.

The LS model, local feature LS model, and GACM have been studied in detail of the previous part, and algorithm experiments have been done using image data [23, 24]. By analyzing the characteristics of each method, the anisotropic diffusion algorithm (ADA) is introduced to carry out smooth filtering on the image. Combined with the advantages of local and global minimization algorithm models, this method is used to overcome the shortcomings of linear filtering, improve the image quality, estimate the edge features of the image target, and improve the level set model segmentation intensity changes, complex background, and strong noise interference of the image target [25, 26].

The filter variational method divides two-dimensional space into two one-dimensional spaces for calculation. By finite difference separation, the one-dimensional problem is considered in the direction, then

(6) $$\begin{array}{c} \phi_{i,j}^{k+1}=\phi_{i,j}^{k}+\mu \Delta t\left(c_{1}\phi_{i+1,j}^{n+1}-c_{2}\phi_{i,j}^{n+1}+c_{3}\phi_{i-1,j}^{n+1}\right)+f_{i}, \end{array}$$

in which *c*_1_ = *δ*_*ε*_(*ϕ*)((*w*_*i*,*j*_^*k*^ + *w*_*i*+1,*j*_^*k*^)/2), *c*_2_ = *δ*_*ε*_(*ϕ*)((*w*_*i*−1,*j*_^*k*^ + 2*w*_*i*,*j*_^*k*^ + *w*_*i*+1,*j*_^*k*^)/2), and *c*_3_ = *δ*_*ε*_(*ϕ*)((*w*_*i*,*j*_^*k*^ + *w*_*i*−1,*j*_^*k*^)/2).

Similarly, consider the one-dimensional problem in the *y* direction using a similar method and then take the average, using the following method:

(7) $$\begin{array}{c} \left(I-2\Delta {tA}_{l}\left(\Phi^{k}\right)\right)\Phi_{l}^{k+1}=\Phi^{k}+f^{k},\Phi^{k+1}=\frac{1}{2}\overset{2}{\underset{l=1}{\sum }}\Phi_{l}^{k+1},l=1,2, \end{array}$$

in which *I* represents the eigenmatrix and *A*_*l*_ is the tridiagonal matrix.

Figure 3 is an experiment of image segmentation by the anisotropic diffusion level set algorithm.  Figure 3(a) is the initial image.  Figure 3(b) is the pixel enhanced image, and Figure 3(c) is the smooth filtering image. Visually, the boundaries are not particularly obvious in the two initial images, and it is indeed difficult to completely detect the main structure of the image and the details of each area. After enhancement and smoothing, the main information structure of the image is highlighted compared to the original image, but the local details are still not obvious.  Figure 3(d) is based on the feature differentiation calculation of the image. The edges are obvious in the enhanced feature image, especially enhanced local and small structures. By using the method of calculating image differentiation, the evolution function can be designed to guide the local level set model to accurately capture the regional features of the image. The image features processed by the improved model are very similar to high-pass filtering, and it can be observed in the experimental results that the model has enhanced the main boundary features of the target. From the medical image experiments, the transverse axis, gray matter, and white matter are not very clear in the MR brain image by filtering variational method to calculate. But according to the image smoothing effect, subject characteristics have been highlighted, and the target structure is not affected through the calculation of the additive variational method.

## 4. Experiment and Analysis

In this paper, the anisotropic diffusion filtering variational algorithm is compared with the local feature LS and global feature LS. According to the experimental results, when the segmentation target has noise, low contrast, and uneven intensity distribution, the proposed model can better detect the target within the image range in this paper. The following experiments are carried out from these aspects of antinoise ability of the algorithm, ability to detect features, and adaptability of the algorithm in COVID-19 image segmentation for discussion and analysis.

### 4.1. Experiment of Noise Image

Figure 4 is the filter variational level set algorithm's application on the segmentation of noise images. In Figure 4, the application of salt and pepper noise image 0.06 test global minimum variational level set algorithm, from longitudinal coronary segmentation of brain MR image results in the observation, 400 iterations of algorithm after continuous evolution, the convergence of algorithm can be divided noise image target, after denoising smoothing. We see the ideal segmentation results in Figure 4(h). Finally, the segmentation region is highlighted in the differential calculation of the longitude variation. This experiment shows that the improved variational minimization level set algorithm has a very good ability to deal with noise and has a strong adaptability to detect the target data.

### 4.2. Experiment of Homogeneous Image Segmentation

Figure 5 shows an experiment of different segmentation models on a homogeneous single-background composite image target. The experiment shows the CV model, local CV model, and filter variational level set model target image segmentation effect; from experimental observation, three kinds of the model level set have advantages including homogeneous segmentation, contrasting good goals, ideal treatment effect, rapid algorithm convergence, and clear segmentation boundary without any loss of feature.

### 4.3. Multiobjective Segmentation Experiment

Multiphase target involves the distribution of different intensities in the image. There are multiple clear cluster intensity distributions in the image, and each separate target is regarded as a cluster.  Figure 6 shows the experimental results of noisy dual-object images by different algorithms.

In Figure 6, three different models are tested using a two-object composite image. It can be seen that all three models detect two targets. In Figure 6, by contrast, the results of the CV model and the local minimization CV model to obtain the goal of the boundary is not completely smooth, especially in the corner or concave boundaries. The variational global minimization model completely captures the details of the image border, and the energy variational model of the double objective has a better ability than the CV model to adapt the shape change of targets. It shows that the improved level set model achieves good results.

### 4.4. Medical Image Segmentation Experiment

Figure 7 is an experiment using coronal sagittal images of the brain. The experimental algorithms include the CV model, local minimization CV model, and filter variational minimization LS algorithm. We see the result of the experiment of filtering the minimization variational LS model compared with two other kinds of algorithms; it has better capabilities of capture target subject structure. Other than that, the filter variational minimization LS method can well detect the details of the brain gray matter and white matter by additive variational processing and the final segmentation result of the less redundant boundary. Since the three models all initialized images from the middle of the target, the detection effect of details in the middle of the brain image was ideal and detected accurately in gray matter and white matter regions. Their differences mainly focus on the edge of the image. Because the gray intensity variation here is intense in the brain images, the structure topology changes a lot, and the detection of boundary information reflects the adaptability of the model and the stability of the algorithm. Experiments with medical image data show that the model has a good ability to deal with objects with complex topological changes, and the curve evolution ability of the model is better.

### 4.5. MR Sequence Image Segmentation Experiment

Figure 8 shows the experiment of the algorithm segmentation of MR sequence lung images in this paper. The sequence images are 64 layers of lung section images. In order to have a certain typicality and representativeness of the experiment, we select the 6 images with obvious target characteristics for experiment of the algorithm. The target of the lung experimental image is very small and it would be difficult to segment it by a single location, so the idea of global capture is still adopted here. After 600 iterations of the algorithm, the algorithm finally obtains a converged segmented image. From the segmentation effect, the lung abscess lesion was completely segmented, and the pulmonary vascular structure had little influence on the segmentation. Finally, the lung abscess lesion was highlighted through differential calculation, and the structure and details of the target were clearly detected with ideal results.

Experiments on lung sequential slice images show that the algorithm has a higher stability in processing objects than other detection methods and has a stronger quality of image edge segmentation and stronger processing ability for objects with uneven image density and overlapping gray structure.

### 4.6. COVID-19 Image Segmentation Experiment

Figure 9 shows the segmentation of the COVID-19 images. To test the reliability of the proposed model on medical images, CT images from the COVID-19 dataset were used to segment the COVID-19 images. In Figure 9, it can be seen that most of the lesions are located around with a slight advantage in the dorsal lung area. Due to special structural and visual features, it is difficult to distinguish the border of the infected area from the chest wall. As a result, some segmentation models have failed to accurately segment areas of COVID-19 infection and accurately detect medical imaging and COVID-19 in chest images. However, by adding significant information to the proposed model, an accurate segmentation of the infected region can be obtained in the COVID-19 images, as shown in Figure 9(c). As a result, the proposed model perfectly extracts the lungs from contrast and challenging backgrounds, and it turns out that the results are closer to manual segmentation. Comparisons with other models show that the proposed model provides better segmentation results for the images.

## 5. Conclusion

In the paper, we analyzed the relevant level set algorithm model and the improved level set model. Based on the theoretical analysis of the variational algorithm model, we proposed the filter variational minimization level set model. The algorithm has excellent ability to detect heterogeneous density images and multiphase target images. The ordinary CV model and the locally minimized CV model can also process the heterogeneous image and the image with some noise pollution and can segment the main structure and some details of the target, but the accuracy is relatively low. The level set model proposed in this paper can process the piecewise constant density image and get the ideal segmentation result. Compared with other variational models, the proposed filter variational level set model has the best segmentation effect when the image quality is provided with heterogeneous intensity, the image target has background change, or the gray structure has topological change. It is more adaptable to the image structure and has a very good antinoise interference ability.

## Figures and Tables

**Figure 1:** Segmentation effect of low-noise and heterogeneous images.

**Figure 2:** Segmentation of heterogeneous images by GACM.

**Figure 3:** Anisotropic diffusion-filtering variational algorithm enhances image features.

**Figure 4:** Filter variational level set algorithm split noise image.

**Figure 5:** Experiment of homogeneous composite image segmentation.

**Figure 6:** Experiment of noisy dual-object images by different algorithms.

**Figure 7:** Segmentation of medical body data by different models.

**Figure 8:** Segmentation of lung MR sequences by the filtering variational algorithm.

**Figure 9:** COVID-19 image segmentation results.

## Data Availability

Original datasets (brain MR image and MR sequence images of lung abscess) are available in a publicly accessible repository: https://fastmri.med.nyu.edu (fastMRI Initiative). Existing COVID-19 datasets are available in a publicly accessible repository: https://github.com/ieee8023/covid-chestxray-dataset.
